This article has been retracted.

# Modeling of Compulsive Behavior Types of Obsessive-Compulsive Disorder Patients by Using the Data Mining Method

**DOI:** 10.1155/2022/8040622

**Published:** 2022-04-23

**Authors:** Şaban Karayağız, Burcu Oralhan, Zeki Oralhan, Hamza Turabieh, Monirujjaman Khan

**Affiliations:** ^1^Department of Psychology, Nuh Naci Yazgan University, 38090 Kayseri, Turkey; ^2^Department of Business Administration, Nuh Naci Yazgan University, 38090 Kayseri, Turkey; ^3^Department of Electrical Electronics Engineering, Nuh Naci Yazgan University, 38090 Kayseri, Turkey; ^4^Department of Information Technology, College of Computing and Information Technology, Taif University, 11099 Taif, Saudi Arabia; ^5^Department of Electrical and Computer Engineering, North South University, Dhaka, Bangladesh

## Abstract

Data mining is a method that is used to find data that are precise, previously uncertain, and logical values from a comprehensive set of information. Data mining is used as a tool for determining the accuracy of classifications of data obtained in the field of bioinformatics by using different algorithm approaches. In this study, the data mining method was used to classify the accuracy of different algorithms and predict the types of compulsive behavior of patients with obsessive compulsive disorder. Data collected from a total of 164 people, 70 males and 94 females, were analyzed. The age range of the people participating in the study was between 7 and 73, and the calculated mean age was 32.4. Data about sociodemographic characteristics, course of disease, treatments, family histories, obsession, and compulsion types of the participants were collected through data collection instruments. Classification algorithm methods found in WEKA software were chosen to process the data. The effect of the types of obsession on the types of compulsion was determined using regression models. The levels of success of the generated models were compared. The results of the study demonstrated the presence of a moderate positive correlation (.35) between these two variables. According to the coefficient of determination, obsession explained 11% of the variance in compulsion. These findings supported the established hypothesis that the effect of the types of obsession was effective on the types of compulsion.

## 1. Introduction

Obsessive Compulsion Disorder (OCD) is a common, often chronic psychiatric disorder, which begins in order to neutralize certain thoughts at the beginning—thoughts entering the person's mind (intrusive) that are repetitive (obsessive) and that the person cannot control—but which, over time, continues with behaviors or mental actions that are done more intensely than they are meant and are done too much, called compulsions, in which the person cannot prevent himself from doing. According to the 2017 data of the World Health Organization, obsessive compulsive disorder affects about 2 to 3% of the world population. Among the treatments administered, the most common are cognitive behavioral therapy, psychotherapy, and drug therapy. However, 40% of patients do not respond to such treatments [1]. Despite many research studies on the etiology of the disease in recent years, comprehensive knowledge has not yet been established. Retrospectively, they describe the onset of obsessive-compulsion disorder (OCD) by linking to the stressful life events experienced by patients, such as childbearing or pregnancy, significant losses, promotion to a new job/position, sexual problems, and severe physical illnesses [2–4]. The themes of OCD symptoms are usually related to contamination, violence, gender, religion, harming, hoarding, and symmetry [5, 6]. Certain researches [7, 8] have studied the relationships between some types of anxiety and OCD. Major examples of such research include compulsive gambling and compulsive sexual behavior. In their study, [9] have revealed the possible dimensions underlying this disorder by using factor analysis on data they collected from 844 adults with obsessive compulsive disorder. In this way, they have examined the clinical relations and familial and genetic bonds. The results they have achieved have revealed two different factors. They are named as order/control and hoarding/instability. They have concluded that the hoarding/instability factor originates from familial and genetic causes. There is OCD research on familial and genetic factors and gender characteristics [10, 11]. In recent years, another emergent field of OCD research has focused on the idea that animals can also get this disease. Thus, new treatment methods to be put on market can be administered to them first. Also, it is easier to carry out scientific modeling in animal populations due to the very dense animal population. Studies have been conducted to uncover the genetic and neuroanatomical basis of the disease by using the method of animal modeling [1, 12–14]. The findings obtained through this modeling method can also be administered to people due to the similarity of genetic characteristics.

For example, [1] have examined animal models used frequently, according to the genetic, pharmacological, behavioral, and predictive validity of OCD in a current review study they have conducted. The first result they have found is that there are not yet enough data for the administration of the currently used animal models to people. Animal models can be an important approach to examining the genetic and neural mechanisms of OCD. They can also be used to develop new therapeutic options for OCD. Finally, future research on OCD-related neurocognitive deficiencies carried out by using similar animal models can be an important tool to decipher the complex etiology of the disease. By using the animal modeling technique, [15] have shown that the avoidance behavior of mice continues after they are stimulated. This ultimately shows that the striatum is the key to the formation and continuity of the behavior of active harm avoidance.

OCD modeling methods used in humans have been increasing in recent years, although less than animal research [16]. A review study on model creation was carried out by examining an OCD patient who had the fear of catching HIV infection. They observed that the patient developed compulsive behaviors such as handwashing. It was seen based on another research study that people given electric shock based on a mathematical modeling gave up their habits of gambling. This suggests that the learning style of harm avoidance is a trait with a neuroanatomical basis in the striatum.

Health data, including general patient profiles, clinical data, insurance data, and other medical data, are recorded for a number of reasons including legal compliance, public health policy analysis, and research, as well as diagnosis and treatment [17]. The data of millions of patient records are examined in order to analyze such recorded data, to search for and identify similarities between patients, and to create a model. Data mining methods can be implemented in the analysis of such large data repositories to shed light on a wide range of health problems. Data mining of quantitative and qualitative such data has great potential to improve health services quality and reduce the cost of delivery of healthcare services [18]. Discovery of a previously unknown relationship through data mining can help organize data for complex problems, give real-time alerts on exceptions, predict the future in various circumstances and scenarios, and estimate threats and opportunities [19].

Data mining is the process of selecting, discovering, and modeling large amounts of data. This process has become an extremely common activity in all areas of the re-research of medical science. Data mining has helped discover useful hidden patterns from large databases. Typical types of health problems that can be eliminated by data mining techniques can be divided into two main categories, including those eliminated by exploration techniques and those eliminated by predictive techniques [20].

In this study, the types of compulsive behavior of patients with OCD were predicted with using the data mining method. Different algorithms were used for classification. Moreover, the performance of algorithms was evaluated.

## 2. Materials and Methods

People included in the study were retrospectively selected from among the patients admitted to the psychiatric clinic in a private hospital between 2015 and 2018, given that they met the necessary conditions. In this context, the purposeful random sampling method was used for the selection of subjects. Access to a group of sociodemographically rich data in particular was of importance to the purpose of the research.

Sociodemographic characteristics of the participants are shown in Table 1. Of the 164 subjects, 70 (42.7%) were male and 94 (657.3%) were female. With regard to the age of the participants, 13 (7.9%) were between 0 and 18 years old, 101 (61.1%) were between 19 and 35 years old, and 50 (30.5%) were 36 years old or older. Regarding their marital status, 89 (54.3%) were married, and 75 (45.7%) were single. Approximately half of them (*n* = 87, 53.0%) had no children. Of the participants, 66.5% were employed, and 62.8 earned between 0 and 2000 Turkish Liras. In terms of the course of the disease, 104 (63.0%) participants had recurrent diseases, 18.3% had first-time diseases, and 18.3% had chronic diseases. As an additional psychological diagnosis, 85 people (51.8%) were diagnosed to have depression. When the participants' family histories were examined, it was reported that no sign was not observed in the immediate relatives of 52.4% of the participants, in collateral relatives of 8.5% of the participants, and in any relatives of 39% of the participants. The most common types of obsession among the participants were doubt (30.5%), contamination (26.8%), order (11.6%), and harm (10.4%). The compulsive behaviors could be listed as control (43.3%), cleanliness (36.0%), and avoidance (9.1%). The content of the other group in the types of obsession included the sexual, religious, somatic, coupling, hoarding, and symmetry factors, while the content of the other group in the types of compulsion included the praying, asking questions, repeating, accumulating, counting, and correction factors. This is the one of the study that used the data mining method to classify the accuracy of different algorithms and predict the types of compulsive behavior of patients with obsessive compulsive disorder.

### 2.1. Data Mining

Data mining is considered a pattern derived from a much larger arrangement of any unfiltered and unformatted information groups. It provides information types for large informatics teams who use at least one computer software program. A data mining research framework is shown in Figure 1. According to the general concept, data mining is a kind of data acquisition. It involves extractions of information, massive information stacks, storages, and computer use. Complex calculations are used in this method, which allows future events to be achieved as desired by breaking down data. The most important features of information extraction are sample expectations for patterns and behaviors, predictions about precise results, the creation of organized information, and dense information indices in research, databases, and the collection of clusters to find the appropriate data [21, 22].

It allows data mining researchers to make sense of complex datasets, assess possible outcomes, and quickly make informed decisions. Data mining or information extraction has applications in various fields such as science, analysis, pharmaceuticals, trade, and security. Developments in recent years have caused a huge increase in data mining applications.

Final inferences can be drawn by classifying and associating data based on specific analyses [24]. The first step in the data mining process is to understand the work to be done and to state the objectives and the problem. Relationships and trends of people included in research are defined. In the next step, the researcher examines the data collected and compares them with the objectives and results set in the first step. At the same time, the nature of the data is also examined. Next, the data are investigated in a preliminary assessment process to be used in the analysis phases. They are arranged appropriately for modelling. Modelling techniques that are chosen are applied to the organized data to come up with the most appropriate parameters. The quality of the model is tested. In the final step, the generated model is implemented, and the results are assessed. Analysis results are presented in an easy-to-understand way, such as images, charts, or tables. The steps in the data mining process can be summarized as explained above [25].

Today, data mining is used in many areas. It is mostly implemented in areas such as healthcare, education, fraud detection, lie detection, market segmentation, research analyses, criminology investigations, bioinformatics, and market analysis. Different approaches, such as multidimensional data analysis, machine learning, soft computing, and data visualization, are used in data mining in general. Hypothesis tests include many statistical techniques such as clustering, classification, and restructuring. The systems that make up the classification are some of the most widely used tools in data mining. Such systems consist of cases, each of which belongs to one of a few classes and is identified by a fixed set of attribute values. A classifier that can accurately predict the class to which a new case belongs is generated. The classification algorithms that were used in the present study were as follows.

#### 2.1.1. Naïve Bayes

It is one of the fastest statistical classifier algorithms and works based on the individual probability of all the features contained in the sample data. It then accurately classifies them. It is used to predict probabilities of class membership, that is, to predict a probability of a share as to whether it belongs to a particular class. Bayesian classification is based on the Bayes' Theorem. In summary, Naive Bayes is a conditional probability model: Given an example of a problem that will be classified and given an example of a problem represented by an *X* = (*x*_1_, *x*_2_, ⋯, *x*_*n*_) vector representing some *n* properties (variables), this example returns the probabilities. For each of the possible outcomes or classes, *p* is (*C*_*k*_  |  *x*_1_, ⋯, *x*_*n*_).

The problem with the above formulation is that if the number of properties is greater than *n* or if a property can receive a large number of values, then it is impossible to base such a model on probability tables. For this reason, a rearrangement is necessary to make the model more traceable. Bayes' Theorem can be defined as a conditional probability [26].

(1) $$\begin{array}{c} p\left(C_{k}\left|X\right.\right)=\frac{p\left(X\left|C_{k}\right.\right).p\left(C_{k}\right)}{p\left(X\right)}, \end{array}$$

In the formula, *X* is the data with unknown class. *C*_*k*_ is the hypothesis *X* which is a specific class. *p*(*C*_*k*_ | *X*) is the probability of the *C*_*k*_ hypothesis referring to *X*. *p*(*C*_*k*_) is the probability of the hypothesis *C*_*k*_ (prior probability). *p*(*X* | *C*_*k*_) is the probability *X* in the hypothesis *C*_*k*_. *p*(*X*) is the probability *X*.

In other words, the above equation can be written by using the Bayesian probability terminology [27].

(2) $$\begin{array}{c} \text{Posterior}=\frac{\text{prior x likelyhood}}{\text{evidence}}. \end{array}$$

#### 2.1.2. Multilayer Perceptron

It is the most popular network architecture in today's world. Each unit generates an effective weighted sum of its inputs and passes this activation level through a transfer function to generate its outputs. Units are organized in a layered feed-forward topology. The network has a simple input–output model with weights and thresholds. Such networks can model functions that determine the complexity of the function. They are almost complex with their number of layers and the number of units on each of their layers. Key topics in the multilayer perceptron are the design characteristics of the number of hidden layers and the number of units on these layers.

A multilayer perceptron is a nonlinear classifier based on perceptron. A multilayer perceptron (MLP) is a backpropagation neural network that has one or more layers between its input and output layers. The following diagram illustrates a three-layered perceptron network.

#### 2.1.3. J48

The J48 classifier is a simple C4.5 decision tree for classification. It is a controlled classification method. It forms a small binary tree. It is a univariate decision tree. It is an extension of the ID3 algorithm. In this classier, the divide and conquer approach is employed to classify data. It divides the data into a range based on the property value of the value found in the training sample.

Because this approach is range-based and univariate, it does not demonstrate a better performance than the multivariate approach. This decision tree is very useful in predicting values. The J48 accuracy of an accurately classified sample is much higher than other algorithms that are univariate in nature.

#### 2.1.4. JRIP

JRip (RIPPER) is one of the main and most popular algorithms. Classes are examined in incremental sizes, and an initial set of rules for the class are generated through incremental errors. JRip (RIPPER) considers all instances of a particular judgment as a class in the training data and progresses by finding a series of rules. It includes all members of this class. After that, it proceeds to a subsequent class and does the same thing, repeating it until all classes are covered [28]. JRip is an optimized version of IREP [29]. It was introduced by William W. Cohen. Repeated incremental JRip produces error reduction [30].

#### 2.1.5. Random Forest

The random forest classifier proposed by Breiman consists of many individual classification trees (in this study, the number of trees is 10), where each tree is a classifier given a specific weight for the classification output (in WEKA, all trees are given the same weight). Classification outputs from all trees are used to determine the overall classification output created by selecting the mode of all tree classification outputs (the output rated the most) [31].

Random Forest (RF) is a method based on decision trees employing binary division rules for data. In classification problems, the main rules employed to divide data are the Gini index, deviation, and extraction rule [32, 33]. Among these rules, the Gini index, which measures node pollution, is the most commonly used rule [34].

This section may be divided by subheadings. It should provide a concise and precise description of the experimental results, their interpretation, and experimental conclusions that can be drawn.

#### 2.1.6. OneR

The OneR algorithm establishes a single rule for each attribute of training data and then accepts the rule with the lowest error rate. In order to create a rule for an attribute, the most recurrent class should be created for each attribute value. The most repetitive class is the most common class that is seen for that attribute value. This rule is a set of attribute values based on the most repeated class that the attribute is based on [35].

The number of samples of the training data that does not match the binding attribute value in the rule gives the error rate. OneR chooses the rule with the lowest error rate. If two or more rules have the same error rate, the rule is chosen randomly [35].

#### 2.1.7. SMO

Platt's Sequential Minimal Optimization (SMO) [36] is a simple and effective algorithm for solving the second-degree programming problem that occurs in support vector machines. Recently, [37] have suggested that a problem caused by the way SMO holds and updates a single threshold value and recommended two modified versions of SMO that overcome this problem.

Its comparison of benchmarking datasets shows that modified algorithms perform significantly faster than the original SMO in most cases. However, the convergence results in these algorithms have not yet been determined [38].

#### 2.1.8. PART

This is a class in order to establish a PART decision list. It uses the split and divide approach, creates a partial C4.5 decision tree in each iteration, and makes the “best” leaf a rule [35]. It combines the divide-and-conquer strategy with separate-and-conquer strategy of rule learning.

#### 2.1.9. Evaluation Tools

In addition to classification algorithms, evaluation tools are often used. Information gain (IG) is a statistical feature that measures how well a specific attribute distinguishes a training sample based on its target classification. The entropy value is commonly used to determine the exact information gain. Entropy is defined as the impurity of an arbitrary collection of samples that are given [39]. The set *S* of examples is partitioned into the subsets *S*_1_ and *S*_2_. Let there be *k* classes *C*_*i*_, ⋯, *C*_*k*_. Let *P*(*C*_*i*_, *S*) be the proportion of examples in *S* that have class *C*_*i*_. The class entropy of a subset *S* is defined as [40]

(3) $$\begin{array}{c} \text{Entropy}\left(S\right)=-\overset{k}{\underset{i=1}{\sum }}P\left(C_{i},S\right)\log\left(P\left(C_{i},S\right)\right). \end{array}$$

The formula evaluates the worth of an attribute by measuring the information gain with respect to the class. According to the set *S* and the potential binary partition by the given cut value *T* of attribute *A*, the information gain of a cut point is given as the following equation [40]:

(4) $$\begin{array}{c} \text{Gain}\left(A,T;S\right)=\text{Entropy}\left(S\right)-\text{Entropy}\left(A,T;S\right). \end{array}$$

What is described in equation (3) is the expected entropy value and is the sum of each child event entropy. Based on the 4-equation information gain, the InfoGainAttributeEval tool on Weka, which evaluates the property, can be used to select relevant genes and to evaluate factors and events in clinical results. When using the MDL-based differentiation method to parse numerical properties, Ranker, the tool to evaluate factors, is used [23]. A factor is ranked by evaluating its properties in the evaluation tool. In this way, the ranking list and scores of associated factors, especially those of interest, are obtained by using the Ranker method [41, 42].

Data mining is used as a tool for determining the accuracy of classifications of data obtained in the field of bioinformatics by using different algorithm approaches. In this study, data mining techniques were used to predict the types of compulsive behavior of OCD patients by ensuring the classification of the accuracy of different algorithms.

## 3. Results

Classification and cross-validation demonstrate how well the properties will perform in a potential identification process with 10-fold cross-validation. Classification is done by programming the software with a sample of dataset and testing the software with the rest of the data sample. WEKA's property ranking tool was used to identify the strongest individual properties and to list them by effect weight.

The 8 algorithms which yielded the best results from among the algorithms in WEKA software were chosen. In this study, the success rates of the JRIP, J.48, Naive Bayes, PART, Random Forest, Multilayer Perception, ONER, and SMO algorithms were found to be higher than those of the other algorithms. The levels of success of the generated models were compared as shown in Table 2.

When the model was analyzed in terms of run time, JRIP, PART, ONER, Naive Bayes, and J.48 were the algorithms with the least elapsed time. The first four algorithms that provided the best values for all criteria were set in italics in the table. The best results were obtained by using the SMO, ONER, JRIP, and J.48 methods in terms of correct classification rate, kappa statistics. The mean absolute error and the best results in terms of relative absolute error were obtained from the ONER method. Moreover, the worst results in terms of the correctly classified sample rate, Kappa statistics, the mean square root of the errors, and the square root of the relative errors were obtained from the Random Forest algorithm.

A decision tree (Alternating Decision Tree (ADTree)) consists of decision nodes and prediction nodes. Decision nodes indicate an action result. Prediction nodes contain a single number. Alternative decision trees always have prediction nodes as both the root and the leaves. Classification of a record is done by following the paths where each prediction node, and all decision nodes that are visited are correct [43–45]. The decision tree created according to j.45 classification for the determination of types of compulsion is shown in Figure 2. J48, also known as the C4.5 decision tree, results in a decision from the nodes formed by dividing the data over the attribute with the highest information gain [46–48]. It is a derivative of the ID3 algorithm.

When the rules obtained from the decision tree nodes were interpreted, the following were observed.

When the employment status of a patient with the obsession type harm was examined, the patient showed control compulsion if the patient was not employed and avoidance compulsion if the patient was employed. A patient with the obsession type contamination showed a cleanliness compulsion. A patient with the obsession type order showed a control compulsion. A patient with the obsession type doubt showed a control compulsion. For a patient with the obsession type “other,” the patient's income status was checked. If the income level was above 2001 Turkish Liras, the patient showed one of the other compulsion factors. If the income level was between 0 and 2000 Turkish Liras, the course of the disease was examined. If the course of the disease was in the first case, the family history was examined. If the family history was immediately relative, gender was taken into consideration. If the person was a female, control compulsion was observed, and if the person was male, cleanliness compulsion was observed. If the family history was collateral relative, cleanliness compulsion was observed, and if there was no sign, avoidance compulsion was observed. When we examined the course of the disease again, if it was chronic, other compulsion was observed. If the course of the disease was recurrent, the gender status was examined. If the person was a female, her marital status was considered. If the person was single, she would be observed to have one of the other compulsion factors, and if married, she was observed to have cleanliness compulsion. If the person was male and was single according to his marital status, he was observed to have cleanliness compulsion. And if he was married, then he was observed to have other compulsion.

In the literature, the five variables that were most effective in the course of the disease were examined by using the Random Forest model, taking into consideration the course of the disease in two groups, chronic and repeated, excluding patients who did not show signs. The decision tree was found to have a correct classification rate of 72.83%. According to the decision tree, patients showing chronic path were those who had a family history with their immediate family, younger than 35 years of age, married, male patients.

Classification and cross-validation determine how well the data properties will perform in a potential identification process. WEKA's property ranking tool was used to identify the strongest individual properties and to list them by effect weight. In this respect, the normalized scores of the variables affecting the types of compulsion are presented in Table 3.

According to WEKA ranker analysis, the type of compulsion was observed to be affected by factors such as obsession type (79%), family history (7%), course of the disease (4%), employment (2%), children (1%), and other factors. In the present study, the hypothesis created for the effect of the types of obsession on the types of compulsion was established as follows.

H1: There is a correlation between obsession factors and compulsion factors.

The correlation between the obsession factors and the compulsion factors was tested by using chi-square analysis, and the correlation coefficient was found to be .345 (*r* = .345, *p* < .001); according to the coefficient of determination, obsession explained 11% of the variance in compulsion. In other words, there was a moderate correlation between the obsession and compulsion factors.

## 4. Discussion and Conclusion

Development and implementation of large data repositories of patient-specific clinical, medical, and health data created during patient encounters at the time of routine conduct of healthcare services have been limited, until recently, to static uses of utilization management, quality assurance, and cost management. These repositories, which focus on reducing medical errors through evidence-based health management, are subjected to more complicated analyses using data mining techniques. These techniques provide a new perspective on the healthcare service process with the help of created decision support systems for a number of events and offer countless opportunities to perform in-depth analysis of data. In the future, we will see not only that the use of data mining techniques in health services will increase but also that such systems will be integrated into health intelligence and health organization strategies. In this way, quality targets can be improved, and costs can be reduced.

In many studies examining the diagnosis, treatment and clinical course of OCD, many factors such as the relationship between obsession and compulsion, their prevalence, and their relationships with sociodemographic factors have been examined. When the recovery rates are examined in general, it is observed that symptoms of 20 to 30% of patients have a pronounced improvement, and in 40 to 50%, moderate improvement is observed in symptoms; and in 20–40% of patients, symptoms remain the same or worsens [49]. Current studies and guidelines [50] have given information about the course and prognosis. However, no studies could be found in the literature that examines in detail factors affecting the course of the disease, such as gender, employment, income, and family history and how such factors interact with the OCD process. The decision tree diagram obtained based on data mining addresses this missing point in the literature. Patient-related data that the clinician can obtain even at the first interview by examining the decision tree will shed light on the possibility of chronicity or renewal of the disease. In this way, the clinician will be able to evaluate the treatment schemes of patients in the first episode of the disease and consider binary approaches during pharmacotherapy and psychotherapy processes. And perhaps, in the light of the new studies supporting this study, treatment algorithms and steps can be revised in the process. New schemes of how to approach patients with a high probability of chronicity or renewal of the disease may be identified.

By these definitions, patient-specific methods can be developed within the methods that can be handled in the psychotherapy of OCD. If the potential of a patient's disease is high compared to the decision tree, SSRIs used in primary care can be added directly to double treatment by adding antipsychotic treatments used in the treatment of augmentation and can compensate for the loss of time and may be compensated for pharmacotherapy and OCD-resistant patients, or in patients who cannot take medication. Applied treatment methods such as TMS can be applied from the beginning of the treatment in a situation where the potential of the disease is shown according to the decision tree.

## Figures and Tables

**Figure 1:** Data mining research framework [23].

**Figure 2:** Decision tree of result.

**Table 1:** Sociodemographic characteristics of the participants.

Variable		CODE	Frequency	Percent	Cumulative percent
Gender	Female	1	94	57.3	57.3
	Male	2	70	42.7	100.0
	Total		164	100.0	

Age	0-18	1	13	7.9	7.9
	19-35	2	101	61.6	69.5
	Up to 36	3	50	30.5	100.0
	Total		164	100.0	

Marital status	Single	1	75	45.7	45.7
	Marriage	2	89	54.3	100.0
	Total		164	100.0	

Child	No	1	87	53.0	53.0
	Yes	2	77	47.0	100.0
	Total		164	100.0	

Occupation	Employed	1	109	66.5	66.5
	Unemployed	0	55	33.5	100.0
	Total		164	100.0	

Income	0-2000	1	103	62.8	62.8
	Up to 2001	2	61	37.2	100.0
	Total		164	100.0	

Disease_his	First	1	30	18.3	18.3
	Chronic	2	30	18.3	36.6
	Repetitive	3	104	63.4	100.0
	Total		164	100.0	

Family_his	(1) Degree relative	1	86	52.4	52.4
	(2) Degree relative	2	14	8.5	61.0
	No feature	3	64	39.0	100.0
	Total		164	100.0	

Obsession	Damage	1	17	10.4	10.4
	Contamination	2	44	26.8	37.2
	Order	3	19	11.6	48.8
	Doubt	4	50	30.5	79.3
	Other	5	34	20.7	100.0
	Total		164	100.0	

Compulsive	Cleaning	1	59	36.0	36.0
	Avoidance	2	15	9.1	45.1
	Checking	3	71	43.3	88.5
	Other	4	19	11.6	100.0
	Total		164	100.0	

**Table 2:** Comparison of results of the generated models.

Classifier	Time taken to build model	Correctly classified instances	Kappa statistic	Mean absolute error	Root mean squared error	Relative absolute error	Root relative squared error
JRIP	*0.00*	*62.19%*	*0.387*	0.267	*0.377*	80.89%	*93.71%*
J.48	*0.00*	*60.98%*	*0.390*	*0.247*	*0.384*	*74.40%*	*94.54%*
Naive Bayes	*0.00*	57.92%	0.345	0.264	*0.366*	79.58%	*90.10%*
PART	*0.00*	56.09%	0.329	*0.250*	0.408	*75.36%*	100.49%
Random Forest	*0.04*	55.48%	0.316	0.255	0.387	77.06%	95.17%
Multilayer Perception	0.44	51.82%	0.255	*0.255*	0.442	*76.89%*	108.79%
ONER	*0.00*	*63.41%*	*0.464*	*0.182*	0.427	*55.11%*	105.14%
SMO	0.04	*65.24%*	*0.471*	0.299	*0.381*	90.16%	*93.82%*

**Table 3:** Scores of the variables affecting the types of compulsion.

Variable	Rank	Normalized
10 obsession	0.479	0.793
9 family_his	0.044	0.073
7 disease_his	0.027	0.044
5 occupation	0.016	0.027
4 child	0.009	0.014
6 income	0.009	0.014
2 age	0.007	0.012
1 gender	0.007	0.012
3 marital status	0.006	0.010
Total	0.604	1.000

## Data Availability

The copyright of the data used in this paper belongs to TMS Clinic and Nuh Naci Yazgan University. So it cannot be disclosed without authorization.
